# Identification and Validation of a Novel Prognostic Gene Model for Colorectal Cancer

This article has been retracted.

**DOI:** 10.1155/2022/9774219

**Published:** 2022-07-25

**Authors:** Yan Meng, Rulin Zhou, Zhizhao Lin, Qun Peng, Jian Ding, Mei Huang, Yiwen Li, Xuxue Guo, Kangmin Zhuang

**Affiliations:** ^1^Guangdong Provincial Key Laboratory of Gastroenterology, Department of Gastroenterology, Nanfang Hospital, Southern Medical University, Guangzhou, Guangdong, China; ^2^Huiqiao Medical Center, Nanfang Hospital, Southern Medical University, Guangzhou, Guangdong, China

## Abstract

**Aims:**

Colon cancer (CRC), with high morbidity and mortality, is a common and highly malignant cancer, which always has a bad prognosis. So it is urgent to employ a reasonable manner to assess the prognosis of patients. We developed and validated a gene model for predicting CRC risk.

**Methods:**

The Gene Expression Omnibus (GEO) database was used to extract the gene expression profiles of CRC patients (*N* = 181) from GEO to identify genes that were differentially expressed between CRC patients and controls and then stable signature genes by firstly using both robust likelihood-based modeling with 1000 iterations and random survival forest variable hunting algorithms. Cluster analysis using the longest distance method was drawn out, and Kaplan–Meier (KM) survival analysis was used to compare the clusters. Meanwhile, the risk score was evaluated in three independent datasets including the GEO and Illumina HiSeq sequencing platforms. The corresponding risk index was calculated, and samples were clustered into high- and low-risk groups according to the median. And survival ROC analysis was used to evaluate the prognostic model. Finally, the Gene Set Enrichment Analysis (GSEA) was performed for further functional enrichment analyses.

**Results:**

A 10-gene model was obtained, including 7 negative impact factors (SLC39A14, AACS, ERP29, LAMP3, TMEM106C, TMED2, and SLC25A3) and 3 positive ones (CNPY2, GRB10, and PBK), which related with several important oncogenic pathways (KRAS signaling, TNF-*α* signaling pathway, and WNT signaling pathway) and several cancer-related cellular processes (epithelial mesenchymal transition and cellular apoptosis). By using colon cancer datasets from The Cancer Genome Atlas (TCGA), the model was validated in KM survival analysis (*P* ≤ 0.001) and significant analysis with recurrence time (*P* = 0.0018).

**Conclusions:**

This study firstly developed a stable and effective 10-gene model by using novel combined methods, and CRC patients might be able to use it as a prognostic marker for predicting their survival and monitoring their long-term treatment.

## 1. Introduction

Colorectal cancer (CRC) is a common malignance worldwide [1, 2]. Patients are usually diagnosed with advanced stage and experience metastatic recurrences even after curative resection. Despite the development of combination therapy strategies for CRC, the overall 5-year survival rate remains low in advanced-stage CRC patients [3].

Carcinogenesis in CRC is a multistep and multifactor process involving genes and epigenetics, and genes that control tumor growth, such as oncogenes or tumor suppressor genes, are activated or inactivated [4]. The recent identification of novel biomarkers and therapeutic targets in CRC has improved the diagnosis and treatment of this disease. However, because of the heterogeneity of this cancer, single biomarkers are limited by poor efficacy. Thus, it would be more beneficial for clinical strategies to identify how the genetic profile of colorectal carcinoma influences prognosis, as well as the accurate risk assessment based on genetic screening [5].

Since the development of bioinformatics, genomic analysis of malignant tumors has become a helpful tool for identifying potential cancer biomarkers [6]. Biomarkers discovered by microarray analysis have good potential for the prediction of clinical outcomes and survival, as well as for the classification of different subtypes. In recent years, studies aimed at establishing proportional hazard models constituted a key step in bioinformatics analysis [7, 8]. A series of methods for screening potential prognostic genes have been developed, including random survival forest variable hunting algorithms and robust likelihood-based survival modeling, among others [9, 10]. However, although these two models have been reported as useful tools in the model construction of CRC, previous studies in this field are mainly based on a single prognostic statistical method, with few studies using two or more prognostic statistical methods in the field of CRC [11–13].

In this study, genomic expression profiles of CRC were analyzed to determine the genes most strongly associated with prognosis. We firstly combined prognostic methods by using both RSFVH and the robust likelihood-based survival model to establish a novel hazard prognostic model. After integrated analysis, a 10-gene expression signature was identified as a novel prognostic model for CRC. The CRC dataset from TCGA was used to determine the stability and effectiveness of this novel hazard model, and this could be used to identify CRC patients with a high mortality risk. In addition to serving as a prognostic signature for CRC patients and monitoring long-term treatment outcomes, a stable and effective 10-gene model may also serve as an indicator for long-term survival, which will provide a reference for clinicians to choose treatment ways for CRC patients.

## 2. Materials and Methods

### 2.1. Source and Processing of Data

Microarray gene expression profiles of GSE41258 were used as a training dataset and downloaded from the GEO database. Firstly, 181 in situ tumor samples from patents with a survival time of >1 month were selected to reduce analytical error caused by extreme conditions after clinical data sorting of these samples. Then, data normalization was performed by log_2_ transformation. TCGA CRC data from Illumina HiSeq and Illumina GA were used as test datasets.

A multistep strategy for identifying CRC prognostic models was diagrammed in Figure 1, summarizing results of each step.

### 2.2. Differential Analysis of Prognostic Genes

Genes with significant changes and differential expression were selected as follows: (1) the total median and variance of all expression levels were calculated from the GEO dataset; (2) the average expression level of selected genes was more than 20% of the average expression level of all genes.

Univariate Cox regression analysis was performed for differentially expressed genes. Genes with differential expression at *P* < 0.05 were selected as significant prognostic genes.

### 2.3. Data Processing

The selected genes were further screened to simplify the constructed prognostic model and to increase the reliability of the model. Random forest-based and robust likelihood-based survival modeling was performed, among which the common genes were selected as feature genes.

### 2.4. Random Forest-Based Survival Modeling

A prognostic random forest variable hunting algorithm, which is an efficient and accurate model, was used for selecting event-specific variables and estimating the cumulative incident function. Based on the prognostic information, the cumulative incidence was calculated and a random forest composed of decision trees was constructed. In addition, we identified variables with a significant impact on prognosis by calculating the prediction error for the proposed ensemble estimators and variable selection and the distance between the first node and the root node in the decision tree [14].

### 2.5. Robust Likelihood-Based Survival Modeling

Another survival model, the robust likelihood survival model, was used to select significantly expressed genes by using rbsurv in R Language as follows:

1. A random sample distribution was used to divide samples into two sets, including a training set with 1/3 of samples and the validation set with 2/3 of the samples
2. Then, 10 log likelihood was used to select the most frequent gene combinations. Genes with the greatest mean log likelihood were selected for further analysis. The next best gene was identified by evaluating all two-gene models, and the ideal gene with the largest mean log likelihood was selected
3. The procedure described above was repeated 1000 times [15–19]

### 2.6. Clustering Analysis and Correlation Analysis of Prognostic Genes

According to the expression of 10 common genes obtained using the two screening models, each sample was divided into two groups by unsupervised hierarchical clustering to verify the effect of the selected genes on prognosis. Briefly, Euclidean distance was calculated with the formula *d*(*AB*) = sqrt [∑((*a*[*i*] − *b*[*i*])^2^)] to detect the distance between samples. The longest distance method (the longest distance method builds a distance matrix and sets the initial new class by using the farthest distance between samples and new classes as the distance) was used as the clustering method [20].

To identify prognostic differences in samples after classification, Kaplan–Meier survival analysis was performed. Simultaneously, Pearson's correlation analysis was used to test the correlation among feature genes.

### 2.7. Construction of the Prognostic Model

A prognostic index linear model was used to construct a prognostic risk model of the 10 feature genes based on Cox proportional hazard regression. The basic form of this model is PI (risk score) = *β*_1_*X*_1_ + *β*_2_*X*_2_ + ⋯⋯+*β*_*m*_*X*_*m*_, in which *β* indicates the regression coefficients for each gene and *X* indicates the gene expression profile [21]. Therefore, the PI value is an indicator of the prognosis of patients, with a higher level representing a greater risk and poorer prognosis of patients.

### 2.8. Validation of the Prognostic Model

In order to validate the robustness of the novel risk score model described above, three independent datasets were used to evaluate the risk score, including the GEO, Illumina HiSeq, and Illumina GA sequencing platforms. The corresponding risk index was calculated, and samples were clustered into high- and low-risk groups according to the median. KM survival analysis was performed to compare the prognosis between two indicated groups.

To avoid overfitting caused by sample heterogeneity, resampling was performed, and 80% of the samples were randomly selected. After dividing the selected samples into high- and low-risk groups, Kaplan–Meier survival analysis was performed and the steps were repeated 500 times. *P* values of <0.05 were considered to indicate a significant difference.

### 2.9. Survival ROC of the Prognostic Model

ROC curves reflect the accuracy of continuous variables for determining dependent variables under different criteria, where the AUC reflects the judgmental value of the independent variables. According to the residual function of two variables, the survival ROC curve transforms the prognostic information into the dependent variable of the ROC curve, representing the prognostic judgmental value of independent variables. A higher AUC indicates a more accurate prognostic prediction of the index [22].

### 2.10. Functional Enrichment Analyses

In this study, a high-risk group and a low-risk group were formed based on risk scores. Genes (GSE: 19820, tcga-Hiseq: 19474, and tcga-ga: 17972) were enrolled into the GSEA process. Three types of gene sets were used in this study. Hallmark and KEGG gene sets were downloaded from MSigDB (http://www.gsea-msigdb.org/gsea/downloads.jsp). GSEA was performed by R “fgsea” package. Gene sets with normalized *P* value < 0.05 and an absolute normalized enrich score (NES) larger than 1 were considered to be significantly enriched.

### 2.11. Statistical Analysis

As described above, genes with differential expression at *P* < 0.05 were chosen as significant prognostic genes in a univariate Cox regression analysis of the differentially expressed genes. Based on the KM survival analysis, the difference in prognosis between sample groups was identified. Also, Pearson's correlation analysis was used to test the correlation among feature genes. Survival ROC curves of prognostic model were carried out. Gene sets of GSEA with normalized *P* value < 0.05. *P* values of <0.05 were considered statistically significant.

## 3. Results

### 3.1. Sample Selection, Data Sources, and Processing

A total of 19820 genomic expression profiles of 390 CRC patients were selected from GSE41258, and 181 formalin-fixed paraffin-embedded tumor tissues were included. Besides, the validation model was based on TGCA dataset. 364 and 215 were obtained from the Illumina HiSeq and Illumina GA sequencing platforms of TCGA dataset, respectively. The overall flowchart of this work is summarized in Figure 1.

### 3.2. Differential Analysis of Prognostic Genes

12546 differentially expressed genes were identified. At the significance level of univariate Cox regression of the differentially expressed genes above adjusted *P* < 0.05, a total of 1723 significantly prognostic expressed genes were identified (Table 1).

### 3.3. Prognostic Gene Screening

Firstly, 23 prognostic genes were screened using the prognosis random forest variable hunting algorithm from the Gene Expression Omnibus (GEO) data (the parameters were 50 repetitions and 50 iterations), including SLC39A14, AACS, STX18, CNPY2, PSMA5, GRB10, ERP29, LAMP3, TMEM106C, OLR1, NEO1, ALG6, PBK, MTUS1, GRP, SLC39A8, TMED2, SLC25A3, XPO7, HOXC10, PPCS, MLLT11, and SDF4.

Then, 12 prognostic genes were screened as the most frequent gene combinations by one thousand robust likelihood-based survival analysis, including ERP29, TMED2, SLC39A14, AACS, CNPY2, PTHLH, SLC25A3, PBK, LAMP3, CAMSAP2, GRB10, and TMEM106C (Table 2).

Finally, the same genes both enrolled in two screening methods, including SLC39A14, AACS, CNPY2, GRB10, ERP29, LAMP3, TMEM106C, PBK, TMED2, and SLC25A3, were selected as the feature genes using the two methods.

### 3.4. Clustering Analysis and Correlation Analysis of Prognostic Genes

Unsupervised hierarchical clustering was applied to the datasets of the expression profiles of 10 feature genes and samples of the GEO dataset (Figure 2), and two clusters were identified as Cluster 1 and Cluster 2.

Kaplan–Meier survival analyses of Cluster 1 and Cluster 2 (Figure 3(a)) showed significant differences in prognosis between Cluster 1 and Cluster 2 (*P* = 0.001). In addition, according to Pearson's correlation analysis, most of the 10 genes were weakly correlated (Figure 3(b)), demonstrating that 10 genes had less information overlap and low redundancy.

### 3.5. Construction of the Prognostic Model

According to Cox regression survival analysis, the prognostic model was defined as follows: prognostic index (PI, risk score) = (−0.88 × SLC39A14) + (−0.13 × AACS) + (0.01 × CNPY2) + (1.08 × GRB10) + (−0.32 × ERP29) + (−0.49 × LAMP3) + (−1.05 × TMEM106C) + (0.16 × PBK) + (−0.66 × TMED2) + (−0.14 × SLC25A3), suggesting that the higher the expression level of the gene with a positive coefficient, the shorter the average survival time, and the higher the expression level of the gene with a negative coefficient, the shorter the survival time.

In the GEO data, median was taken as the cutoff point and the activation factor of each sample was determined, with 1 representing a positive result and 0 representing a negative result. And sum of scores of ten genes was taken as the extra score.

According to the risk index score of the model, we divided the samples into two groups based on their risk of infection: high risk and low risk with all meaningful risk index segmentation points (≥1, ≥2, ≥3, ≥4…), and KM analysis was carried out (Figure 4). It can be seen from the figure that when the segmentation point was ≥6, *P* value was minimum (*P* = 4.07 × 10^−8^). Therefore, 6 or more was chosen as the optimal segmentation point of the additional model risk index score and the ≥6-gene cluster model was identified as the final model of the 10-gene prognostic feature.

### 3.6. Validation of the Prognostic Model

KM survival analyses of low- and high-risk groups showed significant differences in prognosis from the GEO data (Figure 5(a), *P* ≤ 0.001) and TCGA Illumina HiSeq sequencing platform data (Figure 5(b), *P* = 0.018). There was a significant difference in survival rates between the high-risk and low-risk groups for each dataset.

Resampling and the KM survival analyses were performed to estimate the differences in survival time in 80% of cases selected by 500 random sampling events. The difference in the GEO data of 500 random sampling events and the Illumina HiSeq sequencing platform data of TCGA of 312 random sampling events was significant (100% and 62.4%, respectively), whereas there was no significant difference (78%) in TCGA's Illumina GA sequencing platform data of 78 random sampling events.

### 3.7. Survival Receiver Operating Characteristic (ROC) Curve of the Prognostic Model

The 5-year survival ROC curve was drawn according to the risk index, survival time, and survival status of the three groups. AUC of the GEO data was 0.828 (Figure 6(a)), and that of TCGA Illumina HiSeq sequencing platform data was 0.677 (Figure 6(b)).

### 3.8. Identification of 10-Gene Signature-Associated Biological Pathways and Processes

Gene Set Enrichment Analysis (GSEA) was carried out to identify the signaling pathways associated with associated biological processes; we performed the 10-gene model in both GSE41258 and TCGA Illumina HiSeq and Illumina GA sequencing platforms. We found that the identified gene model positively related with several important oncogenic pathways, including KRAS signaling, TNF-*α* signaling pathway, and WNT signaling pathway, both in training set and validating set (Figure 7, NES > 1, *P* < 0.05). Also, several other cancer-related cellular processes, such as epithelial mesenchymal transition and cellular apoptosis (Figure 7, NES > 1, *P* < 0.05), were positively related to this novel 10-gene model, indicating that the signature might be involved in cancer-related pathways.

## 4. Discussion

CRC is a common digestive tract malignancy with high incidence and mortality. Despite advances in CRC screening and treatment, the high recurrence and metastasis rates of CRC lead to poor outcomes. Therefore, accurate assessment of the prognosis of patients with CRC is important. Despite extensive investigation to identify a gene signature for prognosis in CRC, signatures for use in preclinical and clinical research remain inadequate. As part of this study, we developed and validated a stable and effective prognostic gene model based on 10 genes (SLC39A14, AACS, ERP29, LAMP3, TMEM106C, TMED2, SLC25A3, CNPY2, GRB10, and PBK) that have prognostic properties to evaluate the prognostic risk factors of CRC patients. To confirm the differentially expressed gene signatures extracted from the GEO database (GSE41258), two screening methods, named robust likelihood based survival modeling and random forest variable hunting algorithm, were cooperatively applied. Unsupervised hierarchical clustering and KM survival analysis further confirmed the accuracy and rationality of the selected signatures.

To achieve an advanced molecular classifier and predictors, multivariate survival analysis together with an extra model analysis was used to verify the stability and effectiveness of the model using the independent datasets from GEO and TCGA. The predictive value based on the cohort from TCGA Illumina HiSeq was lower than that based on the GEO cohort, possibly because the data in TCGA are generated by large research teams and are more standardized than GEO. Our analysis showed that the 10-gene clustering model could reliably classify patients from the selected dataset and the additional data into high- and low-risk groups with significant differences in survival time.

The 10 genes identified in this study were previously shown to be differentially expressed in a variety of cancers including CRC. SLC39A14, a divalent cation transporter coding gene, has two splice isoforms with a mutually exclusive exon 4, generating two isoforms: SLC39A14-4A and SLC39A14-4B [23]. Based on an analysis involving 244 colorectal tissue samples, Sveen et al. suggested that the biomarker based on the SLC39A14-exon4B transcript variation may be useful in distinguishing CRC from other colon diseases [24]. Therefore, the development of therapeutic strategies targeting alternative splicing may be effective in CRC. ERP29 plays a key role in the processing of secretory proteins within the endoplasmic reticulum in eukaryotic cells. In colon cancer, this molecule was integrated into a novel panel linked to metastasis and was stratified according to the prognostic risks of CRC, suggesting that the expression of ERP29 is strongly associated with cancer cell's metastasis and disease recurrence [25]. LAMP3, which encodes a type 1 integral membrane protein, has been identified as an upregulated glycoprotein potentially involved in the biological processes of tumorigenesis in CRC [26]. Immunohistochemistry analysis of a tissue microarray indicated that epithelial LAMP3 may be an independent prognostic marker both for CRC and gastric cancer [27]. SLC25A3 is involved in the discrimination of chronic phase from blast crisis chronic myeloid leukemia and therefore may help determine risk-based treatment strategies at diagnosis [28]. However, it has not been identified in CRC until now. Upregulation of TMEM106C expression is associated with poor prognosis in hepatocarcinoma patients, indicating that TMEM106C may serve as a new potential target for gene therapy of this malignancy [29]. TMED2 is significantly upregulated in breast cancer and related to unfavorable outcomes [30]. In the cytosol, AACS catalyzes the synthesis of cholesterol and fatty acids from ketones. This study is the first to show that AACS, TMEM106C, TMED2, and SLC25A3 are associated with CRC as negative impact factors that influence the prognosis of CRC.

CNPY2 may modulate the development of CRC by promoting angiogenesis, cell proliferation, and migration, as well as by inhibiting apoptosis by negatively regulating the p53 pathway. CNPY2 may represent a prognostic indicator for CRC [31]. Serum CNPY2 is considered as a valuable diagnostic biomarker in CRC screening [32]. GRB10, which encodes an adaptor protein, modulates the coupling of multiple cell surface receptor kinases involved in specific signaling pathways. Zhang et al. observed significant upregulation of GRB10 expression among 14 genes involved in the PI3K-Akt signaling pathway in CRC [33]. GRB10 is not only a survival-related gene in CRC but is also implicated in the signaling pathways associated with CRC metastases [34]. Overexpression of the PBK gene has been implicated in tumorigenesis [35]. The expression of PBK/TOPK, as analyzed by immunohistochemistry, may serve as an independent prognostic marker for CRC patients [36]. The functions and roles of these genes in CRC warrant further study, and the significance as essential genes in the 10-gene signature cannot be overstated.

Furthermore, the GSEA showed that expression level of several critical oncogenous pathways, including KRAS signaling, TNF-*α* signaling pathway, and WNT signaling pathway, was positively correlative with the constructed 10-gene model. As a result, these findings may play an important role in developing new targeted anticancer therapies. As novel molecular targets, the 10 prognostic genes may have therapeutic potential.

In summary, the constructed 10-gene expression signature was stable and effective in clustering patients with significant differences in clinical outcomes into high- and low-risk groups. Four of the 10 genes were found to be related to CRC for the first time, which can affect the prognosis of patients. This feature gene model has increased our molecular understanding of CRC and might be of great help for predicting the prognosis of CRC patients.

## 5. Conclusion

In the present study, we developed a 10-gene expression signature of CRC by firstly using two novel bioinformatic statistic methods. Kaplan–Meier survival analyses and ROC curve analyses both identified the efficacy of this novel model, which might be a novel tool for predicting the prognosis of CRC patients. However, the limitation of this study is the lack of clinical practice and validation of the present gene model, which needed to be further developed.

## Figures and Tables

**Figure 1:** Diagram of a multistep scheme to identify gene signatures associated with prognosis in colorectal cancer.

**Figure 2:** Clustering analyses of 10 genes. Each sample is represented by a horizontal axis. A vertical axis on the right side shows the feature genes with Pearson's correlation coefficient. Samples could be grouped into two clusters based on the first categorical attribute of the spreadsheet. The “high risk of CRC” samples are shown in red (Cluster 1) and the “normal” samples are shown in blue (Cluster 2).

**Figure 3:** Analyses of KM survival data on prognostic factors. Kaplan–Meier survival analyses of Cluster 1 and Cluster 2 is shown in (a) and Pearson's correlation analysis of 10 genes is shown in (b).

**Figure 4:** Analyses of KM survival for different clusters. The samples were divided into high-risk and low-risk groups based on the activated impact factors of every sample (≥1, ≥2, ≥3, ≥4,…, >9). And significant *P* value (<0.05) of the corresponding cluster was obtained in KM univariate survival analysis.

**Figure 5:** Kaplan–Meier survival analyses of low- and high-risk groups. (a) GEO data. (b) TCGA Illumina HiSeq sequencing platform.

**Figure 6:** ROC curve of risk index, survival time, and survival status. (a) GEO data. (b) TCGA Illumina HiSeq sequencing platform.

**Figure 7:** GSEA of 10-gene model. Hallmark gene analysis of (a) GEO data, (b) TCGA Illumina HiSeq sequencing platform data, and (c) TCGA Illumina GA sequencing platform data was carried out, and several core carcinogenesis pathways enriched from TCGA Illumina HiSeq sequencing platform data are shown in (d).

**Table 1:** Top 20 significantly differential expression genes.

Gene symbol	Cox *P* value
CAMSAP2	9.92*E* − 08^∗^
AKAP12	3.79*E* − 07
ARHGEF40	1.22*E* − 06
EFNB2	1.34*E* − 06
GRB10	2.13*E* − 06
NDRG1	3.52*E* − 06
MLLT11	4.02*E* − 06
PLAT	4.31*E* − 06
CRABP2	6.94*E* − 06
RHBDF1	7.38*E* − 06
FLRT3	7.52*E* − 06
MAP4K4	1.07*E* − 05
LYPD3	1.37*E* − 05
GPC1	1.53*E* − 05
ANO1	1.55*E* − 05
LAMP5	1.55*E* − 05
GSR	1.57*E* − 05
OLR1	1.77*E* − 05
CRYAB	2.01*E* − 05

^∗^ *E* − :10^−^.

**Table 2:** Survival-associated gene signature screening using forward selection.

Gene	nloglik^∗^	AIC
ERP29	312.45	626.91^∗^
TMED2	310.26	624.51^∗^
SLC39A14	304.43	614.87^∗^
AACS	302.66	613.31^∗^
CNPY2	300.13	610.27^∗^
PTHLH	295.35	602.7^∗^
SLC25A3	295.32	604.65^∗^
PBK	295.32	606.64^∗^
LAMP3	294.68	607.35^∗^
CAMSAP2	289.34	598.67^∗^
GRB10	285.22	592.44^∗^
TMEM106C	282.94	589.87^∗^
GSR	282.38	590.77
ALG6	281.9	591.81
SLC39A8	281.76	593.52
PSMA5	281.26	594.53
TSFM	281.22	596.44
XPO7	279.23	594.46
STX18	276.46	590.92

∗: nloglik: negative log-likelihoods; AIC: Akaike information criteria.

## Data Availability

The data used or analyzed during the present study are available from the corresponding author (Kangmin Zhuang) on reasonable request.
